The article "Does auditory attentional bias determine craving for methamphetamine? A pilot study using a word recognition dichotic listening task" was published in 2022. Journal: Heliyon.

# Does auditory attentional bias determine craving for methamphetamine? A pilot study using a word recognition dichotic listening task

**DOI:** 10.1016/j.heliyon.2022.e11311

**Published:** 2022-10-31

**Authors:** Maryam Kazemitabar, Mohammad Taghi Kheirkhah, Mehran Mokarrami, Danilo Garcia

**Affiliations:** a Yale University School of Medicine, New Haven, CT, United States; b Promotion of Health and Innovation (PHI) Lab, International Network for Well-Being, United States; c Institute for Cognitive and Brain Sciences, Shahid Beheshti University, Tehran, Iran; d Department of Psychology, University of Tehran, Tehran, Iran; e Department of Behavioral Sciences and Learning, Linköping University, Linköping, Sweden; f Centre for Ethics, Law and Mental Health (CELAM), University of Gothenburg, Gothenburg, Sweden; g Promotion of Health and Innovation (PHI) Lab, International Network for Well-Being, Sweden; h Department of Psychology, Lund University, Lund, Sweden; i Department of Psychology, University of Gothenburg, Gothenburg, Sweden

**Keywords:** Methamphetamine craving, Implicit assessment, Attentional bias, Dichotic listening paradigm

## Abstract

**Background:**

Obtaining reliable data under explicit evaluations is one of the most complicated challenges in assessing drug users' status. Respondents are likely to give answers that are to their advantage or deliberately deceitful. Regarding drug use, intense and inevitable drug craving is known as one of the main causes of relapse and treatment failure. As a matter of fact, drug craving is directly correlated to attentional bias toward drug-related stimuli, while drug-related stimuli capture drug users' attention as a result of craving. Most methods for studying selective attention and attentional bias have been developed for visual modality. However, stimuli that capture drug users’ attention are not always visual, they could be auditory.

**Aims:**

We examined if a modified word recognition dichotic listening task discriminated between methamphetamine users and non-users. Moreover, we investigated further the reliability and validity of this new paradigm.

**Methods:**

A total of 30 adult males participated in the study (15 methamphetamine users and 15 non-users). The word recognition dichotic listening task included two stimuli narratives/sequences (one neutral and one methamphetamine-related) that were presented simultaneously via headphones, one stimuli sequence to each ear. The participants were instructed to only pay attention to the neutral stimuli and to ignore the drug-related stimuli. Afterward, participants were asked to indicate in a list which words they recognized from the listening task and responded to the Desire for Drug Questionnaire, which was modified to address methamphetamine craving. In addition, a month after the experiment, we assessed therapy adherence among participants who were methamphetamine users.

**Results:**

Methamphetamine users had a significantly lower performance in the word recognition dichotic task compared to non-users (*t* = 4.30, *p* < .001; Cohen’s *d* = 6.13). Importantly, the average performance on the task was significantly higher among methamphetamine users who continued their treatment one month later compared to those who quitted (*t* = −2.56, *p* < .05; Hedges' *g* = 1.28). Moreover, the intraclass correlation coefficient with 95% interval confidence for the word recognition dichotic listening task scores was excellent (ICC = 0.90) and the scores were significantly correlated with self-reported methamphetamine craving (*r* = −.47, *p* < .001).

**Conclusions:**

The modified word recognition dichotic listening task successfully discriminated between individuals who craved methamphetamine from those who did not. This new paradigm demonstrated high reliability and validity in the present pilot study. Due to the importance of preventing unreliable responses when assessing drug cravings, the current method can be, after further validation, utilized in both research and clinical practices.

## 1 Introduction

In the context of drug use, craving encompasses the amount of desire and inclination to use drugs (Rosenberg, 2009). Various methods have been proposed to measure drug craving, such as measures for drug reinforcement, self-administration, psychophysiological responses, neurobiological responses, self-reports, and cognitive processing (Sayette et al., 2000). However, the process of obtaining explicit answers about drug use and craving is complicated because respondents tend to distort their answers or try to deceive clinicians and researchers (Galić et al., 2016). Moreover, due to financial and practical constraints in clinical settings, the use of more sophisticated methods might not be affordable or feasible. In this context, some researchers have suggested that craving is associated with changes in cognitive processing (for a review, see Field et al., 2009). One way to study cognitive processes related to drug cravings might be to use modified tasks that measure attention and memory (Cox et al., 2006; Nguyen-Louie et al., 2016). Such methods are not only less expensive and more feasible solutions, but also might avoid deceitful responses because implicit reactions are gathered through behavioral methods.

Theoretical models and empirical findings suggest that drug users tend to pay much more attention to addictive substances and their associated cues than to neutral cues (Franken, 2003; Kavanagh et al., 2005; Robinson and Berridge, 1993). For instance, this type of attentional bias toward drug-related cues (Field and Cox, 2008; Rooke et al., 2008) has been found for alcohol (Albery et al., 2015), nicotine (Rehme et al., 2018), cannabis (Alcorn et al., 2019), cocaine (Leeman et al., 2014), and opioids (MacLean et al., 2018). In short, researchers suggest that an implicit association is formed between cues related to drugs and their consequent rewards during drug consumption (Filbey and DeWitt, 2012). This explains why salient stimuli related to drugs capture drug users’ attention, which can then be used to measure craving (Albertella et al., 2019).

Intense and inevitable drug craving is known as one of the main causes of relapse and treatment failure in methamphetamine consumption (Qi et al., 2021), which makes methamphetamine one of the most addictive stimulant drugs. In this context, recent research using different paradigms of selective attention including the *Stroop* (Ghavidel et al., 2020) and *dot-probe* (Zhao et al., 2021), as well as using *visual search* with (Tsai et al., 2021) and without eye-tracking (Huang et al., 2020), have found that stimuli related to methamphetamine did capture users' attention. As a matter of fact, there is a dual relationship between selective attention and attentional bias; methamphetamine-related stimuli capture drug users’ attention as a result of craving (Manning et al., 2019), while methamphetamine craving is directly correlated to attentional bias toward methamphetamine-related stimuli (Field et al., 2009).

Most methods for studying selective attention and attentional bias have been developed for visual modality (Field et al., 2009). However, it should be noted that cues related to methamphetamine (i.e., stimuli that capture users’ attention), and any other type of drug for that matter, are not always visual, they could be auditory. Traditionally, dichotic listening has been used as a paradigm for studying selective auditory attention in which two auditory sequences—typically speech—are presented to the participant simultaneously. One sequence is presented to one ear while another sequence is presented to the other ear. The participant is asked to pay attention to and then report the content presented in one sequence and ignore the other (Eysenck et al., 1987). We argue that this paradigm can provide an implicit approach for measuring attentional bias toward methamphetamine-related cues.

In this study, using methamphetamine-related auditory stimuli, we examined whether methamphetamine users and non-users can be discriminated. Moreover, we further investigated the reliability and validity of this new methodology.

## 2 Methods

### 2.1 Ethical considerations

All procedures in this study were in accordance with the ethical considerations of the World Medical Association Declaration of Helsinki (2013) for human participants. The participants were informed of the purpose of the study, that the study was confidential and voluntary, and that they were free to withdraw from the study without any consequences. The participants who wanted to take part in the study were asked to sign the informed consent form. The informed consent form was provided by the Iranian National Committee for Ethics in Biomedical Research, which was the same entity that approved the present study (protocol nr. IR.SBU.REC.1400.138). In addition, participants were asked to contact the experimenter in case they needed more information or had any concerns.

### 2.2 Power analysis

To ensure a sufficient sample size, we performed a priori power analysis using G∗Power (Faul et al., 2009). Considering a previous relevant study (Fadardi and Ziaee, 2010), significance level, power, and effect size were determined for an independent samples *t*-test. A minimum required sample size of 52 participants was estimated to detect an effect size of Cohen's *d* = .71 at a significance level of *α* = .05 with a power of 1 − *β* = .80.

### 2.3 Participants

Using convenience sampling, a total of 59 adult males, including methamphetamine users and non-users, who fulfilled our initial screening criteria (i.e., proper hearing and recognition memory and clinic eligibility criteria for methamphetamine users) agreed to participate in the study. All participants had normal or corrected hearing. We also assessed participants’ recognition memory to avoid the effect of innate between-group differences in memory performance on the interpretation of our final results. Half of the participants were patients from a methamphetamine rehabilitation center located in Tehran, while the other half were recruited from the general population through an online invitation. Methamphetamine users were required to meet the following criteria: (1) a history of regular drug use for at least three months, (2) no history of diagnosed psychiatric or neurologic conditions other than substance use disorders, (3) not having used other drugs before or at the time of the study, and (4) consent to participate in the study. Inclusion criteria for non-user were as follows: (1) no history of drug use before or during their participation in the study, (2) no history of diagnosed psychiatric or neurologic conditions, and (3) consent to participate in the study. Eight methamphetamine users were not included in the study after initial screening (five due to comorbid psychiatric disorders; two due to using drugs other than methamphetamine; and one due to not understanding the instructions) and four were excluded for not providing sufficient data or outlier responses (i.e., *n* = 12). In the non-user population, 13 individuals were not included in the study after initial screening (four due to a history of diagnosed psychiatric disorders; four due to the use of various drugs; and five others as a result of deviating from the average age of the methamphetamine users) and data from four individuals were excluded due to their missing or outlier responses (i.e., *n* = 17). Hence, a total of 30 individuals were included in the final analyses, 15 methamphetamine users (*M*_*age*_ = 33.60, *SD* = 2.58) and 15 non-users (*M*_*age*_ = 33.93, *SD* = 2.46). The demographic characteristics of the participants are summarized in Table 1. One month after the experiment, we contacted the rehabilitation center to retrieve who of the 15 drug user patients that, on voluntary basis, still continued their methamphetamine cessation therapies (i.e., adherence to their treatment). Figure 1 shows the participant selection and condition allocation for the present pilot study.

**Table 1:** Descriptive characteristics of both samples.

Variable	*N* = 30	*M* (*SD*)	%
Gender			
Male	30		100
Age groups	30	33.76 (2.48)	
Methamphetamine Users	15		50
Non-users	15		50
Handedness			
Right	30		100
Wight			
Methamphetamine Users	15	69.56 (77.49)	
Non-users	15	73.76 (13.73)	
Height	127		
Methamphetamine Users	15	176.94 (10.61)	
Non-users	15	175.23 (11.23)	
Marital status			
Single	12		40
Married	11		36.66
Divorced or separated	7		23.33
Socioeconomic status			
Low	6		20
Middle	21		70
High	3		30
Education			
Illiterate	1		3.33
(High) school	16		53.33
Bachelor's degree	10		33.33
Master's degree	3		10
Consumption methods∗			
Smoking	7		46.66
Snorting	2		13.33
Injection	6		40
Pills	8		53.33
Consumption frequency†			60
Every day	9		20
Nearly every day	3		6.66
3–4 times a week	1		6.66
Two times a week	1		6.66
Once a week	1		

∗ Consumption among some users was through more than one method.

† Patients who consumed methamphetamine less than once a week or irregularly were not included in the study.

**Figure 1:** Participant selection and condition allocation. Note: WRDLT = Word Recognition Dichotic Listening Task.

## 3 Measures

### 3.1 Recognition memory

To screen participants for auditory recognition memory, we used the *Rey Auditory Verbal Learning Test* (Boake, 2000; Lezak et al., 2004). Numerous versions of the test have been translated into different languages (e.g., Ferreira Correia and Campagna Osorio, 2014; Lavoie et al., 2018). Jafari et al. (2010) have standardized the Persian version used in this study, which has shown acceptable reliability and validity in the Iranian context. The test started by letting participants listen to a list of 15 words that were read to them with a frequency of one word per second and then asking them to recall as many words as they could. This process was repeated five times. To interfere with the stimuli of the first list, a new list of 15 words that were semantically or phonetically similar to the words in the first list was presented. To measure auditory recognition memory, a list of 50 words containing the two mentioned lists (*n* = 30) and 20 new words was presented. Participants were asked to indicate whether each one of the 50 words had been on the initial list or not (*yes*/*no*). Past studies show that, among healthy adults, the word recognition mean was 10.64 ± 2.47 (Jafari et al., 2010). Individuals with a recognition memory score that was one standard deviation below the mentioned mean were not included in the study.

### 3.2 Explicit self-report of craving for methamphetamine

By adapting the *Desire for Drug Questionnaire* (Franken et al., 2002), we developed a version that we called the *Desire for Methamphetamine Questionnaire*. In short, with the permission of the original author, the word “heroin” was replaced with the word “methamphetamine” throughout the questionnaire and then translated into Persian. For example, “using heroin would be pleasant now” was changed to “using methamphetamine would be pleasant now.” The modified version of the questionnaire had acceptable internal consistency reliability in the present study (*Cronbach's α* = .73).

### 3.3 Implicit craving for methamphetamine

In order to measure implicit attentional bias to methamphetamine-related auditory stimuli, we modified the dichotic listening paradigm into a task called *word recognition dichotic listening task*. The stimuli included two narrations/sequences, one neutral and the other related to methamphetamine. The sequences were presented simultaneously, one stimuli sequence to each ear, via headphones. A database of neutral and methamphetamine-related words previously developed in Persian (Ekhtiari et al., 2010) was used to generate the narrations. The duration of playing the two narrations was equal (3 min) and included meaningful sentences. However, there was no semantic relationship between the sentences. Both narrations were read by the same person (i.e., a forty-year-old man). The sound was loud enough for an ordinary conversation (60 dB; Chepesiuk, 2005). Participants were requested to ignore the narrations in one ear and to focus on those in the other and were blinded in terms of which narration was heard from which ear. However, they were required to focus on the ear indicated on the screen in front of them, which was always the neutral narration and selected at random at the beginning of the experiment (i.e., blind for the experimenter). Following the presentation of the stimuli, participants were required to perform the word recognition task by indicating (*yes/no*) if the words were present in the narration they were asked to pay attention to (40 trials; 20 familiar and 20 novel words). Lower response accuracy was considered to indicate attentional bias toward methamphetamine-related content. In other words, it was assumed that the lower an individual performs, the greater he/she is distracted by their to-be-ignored ear (i.e., the methamphetamine-related narration). The task was programmed and run using the Psychopy v3.0 software package (Peirce et al., 2022).

## 4 Procedure

After screening the participants for auditory recognition memory, a single-session experiment using the word recognition dichotic listening paradigm was conducted on both groups. Distractions, if any, were removed from the participants' environment before the experiment began, and the participants were asked about the quality and quantity of their last night's sleep. The participants who did not get enough sleep or felt unwell for any reason were asked to return another day. Through verbal instruction, participants were informed that two different narrations will be playing into each ear separately via headphones (Tanaka et al., 2021; Satz, 1986). At the same time, the instructions appeared on the screen in written form. Participants were asked to wear the headphones and listen carefully, for the next 3 min, only to the sound in their ears as indicated on the computer screen in front of them. At random, one ear received the methamphetamine-related narration and the other ear received the neutral narration—half of the participants listened to methamphetamine-related narration in their right ear while the other half listened in their left ear. Participants had to selectively pay attention only to the determined ear which always was the neutral narration and ignore the other ear—participants did not know what they were going to listen to. They were notified that there will be further measurements concerning the narrations and that they needed to remember the words provided to the determined ear. Then, the participants were examined using a word recognition task. The task consisted of a stimulus (word) and two response options (*yes*/*no*) per trial. In each trial, participants were asked to decide whether the word in question had previously been presented in the auditory task. During this stage, no comments or feedback were made on the participants' performance. Trials remained on the screen until the participants responded using the defined keys on the keyboard (“Z” for *yes* and “slash” for *no*).

To investigate the reliability of the task, we examined the individuals’ task performance twice. After 20 min, participants were asked to take part in the same word recognition task again. At the end of the session, they replied to the *Desire for Methamphetamine Questionnaire*. To be able to investigate the predictive criterion validity of the task, one month later, the rehabilitation center was contacted to determine the willingness of patients to voluntarily continue their methamphetamine cessation therapy.

## 5 Data analysis

The data were analyzed in two steps. The first step was performed to compare the differences in attentional bias to methamphetamine-related auditory stimuli between the two groups using an independent samples *t-test*. The second step included analyses to evaluate the reliability and validity of the task used in the experiment. The intraclass correlation coefficient was used to evaluate the test-retest reliability (stability) and the Pearson correlation coefficient and independent samples *t-tes*t were used to evaluate the construct validity (convergent and discriminant, respectively). Finally, an independent samples *t-test* was used to evaluate the predictive criterion validity by comparing the word recognition dichotic listening task scores of users who quit their therapy after one month with the scores of those who continued with their therapy. The effect size was measured for both test and retest measurements using G∗Power v3.1.

## 6 Results

Individuals with different levels of education were matched between the experiment and control group (three with no academic degree, seven with bachelor's, and five with master's degree). Independent samples *t*-tests were conducted to analyze the mean differences in age, recognition memory, word recognition task, methamphetamine craving self-report, and therapy adherence between the groups (see Table 2). Skewness and kurtosis values for all variables were between ±1.96 (Mayers, 2013), therefore, we assumed that the data was normally distributed. In addition, Levene’s test indicated that variances across groups were equal (*p* > .05). Age and recognition memory differences were not significant between groups (*p* > .05), thus suggesting that users and no-user were similar regarding age and memory. In addition, self-reported craving for methamphetamine at baseline, was higher among users compared to non-users (*t* = −16.73, *p* < .001; Cohen’s *d* = 6.12). Thus, validating the allocation of participants in the drug user and non-user groups.

**Table 2:** Independent samples t-tests for means in age, recognition memory, WRDLT-scores, and self-reported craving.

Variable	Group	N	M (SD)	Skewness	Kurtosis	Statistics
Age	Users	15	33.60 (2.58)	0.03	−1.05	*t* = 0.36; *df* = 28; *p* = .72; Cohen's *d* = .13
	Non-users	15	33.93 (2.46)	−0.24	−0.83	
Recognition Memory	Users	15	11.33 (1.54)	−0.78	−0.06	*t* = 0.97; *df* = 28; *p* = .34; Cohen's *d* = .35
	Non-users	15	11.86 (1.45)	−0.37	−0.37	
WRDLT	Users	15	13.20 (1.26)	0.05	−1.00	*t* = 4.30; *df* = 28; *p <* .001; Cohen's *d* = 1.57
	Non-users	15	15.46 (1.59)	0.43	−0.74	
WRDLT-retest	Users	15	11.46 (1.24)	0.47	−0.52	*t* = 3.63; *df* = 28; *p <* .001; Cohen's *d* = 1.33
	Non-users	15	13.46 (1.72)	0.11	−1.38	
Craving Explicit Self-Report	Users	15	56.01 (6.46)	0.17	−0.44	*t* = −16.73; *df* = 28; *p* = .001; Cohen's *d* = 6.12
	Non-users	15	24.26 (3.47)	0.35	−0.29	
WRDLT Follow-up	Quitted	5	10.01 (1.05)	0.71	−0.45	*t* = −2.56; *df* = 13; *p* = .024; Hedges' *g* = 1.28
	Continued	10	12.40 (1.14)	0.40	−0.02	

Note: Age is indicated in years; WRDLT = average performance on the word recognition dichotic listening task; WRDLT-retest = average performance on the retest of the word recognition dichotic listening task; WRDLT Follow-up = average performance on the word recognition dichotic listening task one month later.

To the best of our knowledge, this is the first time a modified dichotic listening task was used to measure implicit attentional bias toward methamphetamine-related stimuli, thus, we found it necessary to investigate its construct validity, reliability, convergent validity, and predictive criterion validity. First, individuals who were methamphetamine users had a significantly lower performance in the word recognition dichotic task compared to non-users (*t* = 4.30, *p* < .001; Cohen’s *d* = 1.57). Thus, showing that our modified word recognition dichotic listening task properly discriminated methamphetamine users from non-users and therefore had good construct validity (see Table 2).

Regarding the test-retest reliability of the word recognition dichotic listening task, the intraclass correlation coefficient with 95% interval confidence was excellent (ICC = 0.90). The significant correlation between the word recognition dichotic listening task scores and the self-reported explicit methamphetamine craving (*r* = −.47, *p* < .001) implied that there was a convergence between these variables (Figure 2).

**Figure 2:** Correlation plot of word recognition dichotic listening task (WRDLT) scores and the self-reported explicit reports of methamphetamine craving.

Finally, we compared the word recognition dichotic listening task scores between drug users who voluntarily continued their therapy against the scores of those who quit after one month. Again, the analysis showed that our modified task had good predictive criterion validity—patients who later quit the therapy had lower performance on the word recognition dichotic listening task one month earlier (*t =* −2.56, *p =* .02; Hedges' *g* = 1.28).

## 7 Discussion

The present study revealed that compared to non-users, methamphetamine users had a lower performance in the word recognition dichotic listening task and higher scores on the explicit self-reports of methamphetamine craving. These results suggested that the craving for methamphetamine can be measured through the modified task of dichotic listening used in this study. To the best of our knowledge, this is the first study that used the dichotic listening paradigm in combination with a word recognition task to measure craving for drugs.

However, the dichotic listening paradigm has been studied in various fields and proved to be a beneficial method due to its high reliability. Westerhausen and Samuelsen (2020), for example, assessed hemispheric dominance for speech processing using the dichotic listening paradigm with test-retest reliability of .91 and .93. In another study, Hugdahl and Hammar (1997) used the dichotic listening paradigm in the assessment of the performance to consonant-vowel syllables under three different attentional instructions, which resulted in test-retest reliability ranging from .61 to .86. Additionally, Parker et al. (2021) evaluated the reliability of an online behavioral laterality battery using a dichotic listening task that yielded relatively high reliability (*r* = .75). In the present study, we also obtained high test-retest reliability (ICC = 0.90) and very large effect sizes (Cohen's *d* = 1.57 and 1.33 for test and retest measurements respectively) (cf. Sawilowsky, 2009). Hence, this indicates the effectiveness of this method in a new field—the measurement of craving for methamphetamine.

The negative correlation between the word recognition dichotic listening task performance and the explicit reports of craving for methamphetamine disclosed that individuals with methamphetamine dependence who acquired lower scores in the task (i.e., higher attentional bias for methamphetamine) had higher levels of craving. Therefore, we argue that the word recognition dichotic listening task is an applicable implicit method to screen individuals’ cravings for methamphetamine. Despite these results, we cannot conclude that all individuals who have acquired lower scores in the word recognition dichotic listening task necessarily are or will be using methamphetamine. Nevertheless, we argue that at the very least they might be prone to use it in case the drug is available to them. After all, craving for methamphetamine is recognized as a main trigger for methamphetamine use (Bruehl et al., 2006).

Aligned with our results, Witkiewitz and Bowen (2010) suggested that participation in therapy sessions is significantly associated with the craving for drugs. That is, those with higher cravings are more susceptible to quitting treatment sessions. In addition, undertreated withdrawal and ongoing craving to use drugs, uncontrolled acute and chronic pain, stigma, and discrimination by hospital staff about their drug use, and hospital restrictions are among the reasons that cause drug users to quit therapy sessions (Simon et al., 2020). In contrast, follow-ups after the termination of therapy sessions, are efficient to prevent future relapses in those who seek treatment (Marks et al., 2020). Moreover, stable employment history, compulsory supervision, existence of a substitute dependence, starting a new relationship, engagement with inspirational groups (de Albuquerque and Nappo, 2018), and multimodal interventions that consider individual, familial, and social vulnerabilities (Darharaj et al., 2017) help to prevent relapse and decrease drug use. The present study suggests that low performance in the dichotic listening task may be an early indicator of patients at risk for relapse, thus, providing implicit insight about who needs to be followed up during and after therapy.

## 8 Limitations, strengths, and recommendations for future studies

The findings obtained in the present study should be interpreted with caution. First, the participants in this study included only males since very few females with substance use disorders are referred to therapeutic and consultation centers in Iran. The reason for this is the more severe cultural and social stigma attached to substance use among Iranian women (Khazaee-Pool et al., 2019). In addition, despite the fact that it might also be applicable and effective for users of other kinds of drugs, this paradigm was applied only to users of methamphetamine due to them being higher in numbers compared to users of other drugs in the targeted clinic. However, it was still difficult to recruit participants, which limited the sample size. In spite of the initial sample size being larger than the estimated minimum, the unexpected drop-out of some participants made the sample size smaller than required. Another limitation is that auditory distraction can be caused by external or internal factors other than the "desired" distractor (i.e., methamphetamine-related content). Controls applied to sample selection and experiment setting, as well as random allocation of stimulus presentation, can partially rule out the involvement of these variables. Despite these limitations, the present pilot study provides adequate preliminary evidence. That being said, we recommend that future studies use the word recognition dichotic listening task method to assess craving for various drugs and with larger sample sizes.

Moreover, we used convenience sampling in this study, which does not allow for generalizability; therefore, the results of the present study are limited to the specific sample we assessed. On the other hand, since we considered the homogeneity of the participants, our results have clearer generalizability relative to conventional convenience sampling (Jager et al., 2017). Researchers who are interested in trying this method are recommended to use a probability sampling method. Another issue to manage in future studies is that, alongside the desire for the drug, attentional bias may also occur as a consequence of aversion (Belova et al., 2007). Thus, a person may find methamphetamine-related stimuli salient and distracting because they hate the drug. In other words, although the method developed in this study can properly discriminate the level of craving between individuals who currently use the drug and those who do not; there is a possibility that non-users, whose relatives or partners are using the drug, might be biased toward or against methamphetamine-related stimuli. Hence, understanding how at-risk individuals will respond to the word recognition dichotic listening task requires further studies.

One way or another, the current and future challenges of the 21st century, require that we identify methods to measure and understand what makes people crave drugs, such as methamphetamine. During stressful situations, it is harder for people to make the healthy self-directed choices that are necessary to be resilient but easier to start drinking alcohol or taking drugs in order to calm the nervous system (Wong and Cloninger, 2010). Regarding measurement, implicit methods are among the most reliable evaluation methods, especially when the respondents tend to deceive the examiner or have bias regarding the construct under measurement. The current method is a non-invasive, easy-to-use, and feasible paradigm to discriminate between individuals with and without craving for methamphetamine, and can be utilized for monitoring individuals prone to engage in methamphetamine use and regarding their treatment adherence. Additionally, this method can be used to investigate craving for other drugs and other sensitive constructs such as political views, criminal issues, etcetera (Nosek and Hansen, 2008).

## 9 Conclusion

This study provides the first preliminary evidence that our dichotic listening paradigm can be used to measure craving among methamphetamine users. We found that by using a modified dichotic listening task, methamphetamine users and non-users could be discriminated based on their implicit attentional biases toward methamphetamine-related stimuli. Also, the correlation between implicit attentional bias and explicit self-reports of craving for methamphetamine showed that auditory implicit attentional bias is an indicator of drug craving. Moreover, the reliability and validity analyses revealed that our word recognition dichotic listening task is suitable for measuring craving for methamphetamine in both research and clinical settings.

## Declarations

### Author contribution statement

Maryam Kazemitabar: Analyzed and interpreted the data; Wrote the paper.

Mohammad Taghi Kheirkhah: Conceived and designed the experiments; Performed the experiments; Wrote the paper.

Mehran Mokarrami: Performed the experiments; Analyzed and interpreted the data; Wrote the paper.

Danilo Garcia: Conceived and designed the experiments; Wrote the paper.

### Funding statement

This research did not receive any specific grant from funding agencies in the public, commercial, or not-for-profit sectors.

### Data availability statement

Data will be made available on request.

### Declaration of interest’s statement

The authors declare no conflict of interest.

### Additional information

No additional information is available for this paper.

## References

[bib1] Albertella L., Le Pelley M.E., Chamberlain S.R., Westbrook F., Fontenelle L.F., Segrave R., Lee R., Pearson D., Yücel M. (2019). Reward-related attentional capture is associated with severity of addictive and obsessive-compulsive behaviors. Psychol. Addict. Behav..

[bib2] Albery I.P., Sharma D., Noyce S., Frings D., Moss A.C. (2015). Testing a frequency of exposure hypothesis in attentional bias for alcohol-related stimuli amongst social drinkers. Addict. Behav. Rep..

[bib3] Alcorn J.L., Marks K.R., Stoops W.W., Rush C.R., Lile J.A. (2019). Attentional bias to cannabis cues in cannabis users but not cocaine users. Addict. Behav..

[bib4] Belova M.A., Paton J.J., Morrison S.E., Salzman C.D. (2007). Expectation modulates neural responses to pleasant and aversive stimuli in primate Amygdala. Neuron.

[bib5] Boake C. (2000). Edouard Claparede and the auditory verbal learning test. J. Clin. Exp. Neuropsychol..

[bib6] Bruehl A.M., Lende D.H., Schwartz M., Sterk C.E., Elifson K. (2006). Craving and control: methamphetamine users’ narratives. J. Psychoact. Drugs.

[bib7] Chepesiuk R. (2005). Decibel hell: the effects of living in a Noisy World. Environ. Health Perspect..

[bib8] Cox W.M., Fadardi J.S., Pothos E.M. (2006). The addiction-stroop test: theoretical considerations and procedural recommendations. Psychol. Bull..

[bib9] Darharaj M., Habibi M., Kelly A.B., Edalatmehr Z., Kazemitabar M. (2017). Predisposing personality traits and socio-familial factors of tendency toward substance use among soldiers. J. Subst. Use.

[bib10] de Albuquerque R.C.R., Nappo S.A. (2018). Reasons to crack consumption relapse. Users’ perspective. J. Bras. Psiquiatr..

[bib11] Ekhtiari H., Alam-Mehrjerdi Z., Hassani-Abharian P., Nouri M., Farnam R., Mokri A. (2010). Examination and evaluation of craving-inductive verbal cues among Persian-speaking methamphetamine Abusers. Adv. Cogn. Sci..

[bib12] Eysenck M.W., MacLeod C., Mathews A. (1987). Cognitive functioning and anxiety. Psychol. Res..

[bib13] Fadardi J.S., Ziaee S.S. (2010). A comparative study of drug-related attentional bias: evidence from Iran. Exp. Clin. Psychopharmacol.

[bib14] Faul F., Erdfelder E., Buchner A., Lang A.-G. (2009). Statistical power analyses using G∗Power 3.1: tests for correlation and regression analyses. Behav. Res. Methods.

[bib15] Ferreira Correia A., Campagna Osorio I. (2014). The rey auditory verbal learning test: Normative data developed for the venezuelan population. Arch. Clin. Neuropsychol..

[bib16] Field M., Cox W.M. (2008). Attentional bias in addictive behaviors: a review of its development, causes, and consequences. Drug Alcohol Depend..

[bib17] Field M., Munafò M.R., Franken I.H.A. (2009). A meta-Analytic investigation of the relationship between attentional bias and subjective craving in substance Abuse. Psychol. Bull..

[bib18] Filbey F.M., DeWitt S.J. (2012). Cannabis cue-elicited craving and the reward neurocircuitry. Prog. Neuro Psychopharmacol. Biol. Psychiatr..

[bib19] Franken I.H.A. (2003). Drug craving and addiction: integrating psychological and neuropsychopharmacological approaches. Prog. Neuro Psychopharmacol. Biol. Psychiatr..

[bib20] Franken I.H.A., Hendriks V.M., Van den Brink W. (2002). Initial validation of two opiate craving questionnaires: the obsessive compulsive drug use scale and the desires for drug questionnaire. Addict. Behav..

[bib21] Galić Z., Bubić A., Kovačić M.P. (2016). The Wiley Handbook of Personality Assessment.

[bib22] Ghavidel N., Khodagholi F., Ahmadiani A., Khosrowabadi R., Asadi S., Shams J. (2020). Frontocingulate dysfunction is associated with depression and decreased serum PON1 in methamphetamine-dependent patients. Neuropsychiatric Dis. Treat..

[bib23] Huang Y., Liu Z., Ji H., Duan Z., Ling H., Chen J., Ding X. (2020). Attentional bias in methamphetamine users: a visual search task study. Addict. Res. Theor..

[bib24] Hugdahl K., Hammar Å. (1997). Test-retest reliability for the consonant-vowel syllables dichotic listening paradigm. J. Clin. Exp. Neuropsychol..

[bib25] Jafari Z., PS M., Zandi T., AAK K., Malayeri S. (2010). Iranian version of the rey auditory verbal learning test: a validation study. Payesh. Health Monitor.

[bib26] Jager J., Putnick D.L., Bornstein M.H. (2017). II. More than just convenient: the scientific merits of homogeneous convenience samples. Monogr. Soc. Res. Child Dev..

[bib27] Kavanagh D.J., Andrade J., May J. (2005). Imaginary relish and exquisite torture: the elaborated intrusion theory of desire. Psychol. Rev..

[bib28] Khazaee-Pool M., Pashaei T., Nouri R., Taymoori P., Ponnet K. (2019). Understanding the relapse process: exploring Iranian women’s substance use experiences. Subst. Abuse Treat. Prev. Pol..

[bib29] Lavoie M., Bherer L., Joubert S., Gagnon J.F., Blanchet S., Rouleau I., Macoir J., Hudon C. (2018). Normative data for the rey auditory verbal learning test in the older French-Quebec population. Clin. Neuropsychol..

[bib30] Leeman R.F., Robinson C.D., Waters A.J., Sofuoglu M. (2014). A critical review of the literature on attentional bias in cocaine use disorder and suggestions for future research. Exp. Clin. Psychopharmacol.

[bib31] Lezak M., Howieson D., Loring D., Fischer J. (2004).

[bib32] MacLean R.R., Sofuoglu M., Brede E., Robinson C., Waters A.J. (2018). Attentional bias in opioid users: a systematic review and meta-analysis. Drug Alcohol Depend..

[bib33] Manning V., Garfield J.B.B., Mroz K., Campbell S.C., Piercy H., Staiger P.K., Lum J.A.G., Lubman D.I., Verdejo-Garcia A. (2019). Feasibility and acceptability of approach bias modification during methamphetamine withdrawal and related methamphetamine use outcomes. J. Subst. Abuse Treat..

[bib34] Marks L.R., Munigala S., Warren D.K., Liss D.B., Liang S.Y., Schwarz E.S., Durkin M.J. (2020). A comparison of medication for opioid use disorder treatment strategies for persons who inject drugs with invasive bacterial and fungal infections. JID (J. Infect. Dis.).

[bib36] Mayers A. (2013).

[bib37] Nguyen-Louie T.T., Buckman J.F., Ray S., Bates M.E. (2016). Drinkers’ memory bias for alcohol picture cues in explicit and implicit memory tasks. Drug Alcohol Depend..

[bib38] Nosek B., Hansen J. (2008). The associations in our heads belong to us: searching for attitudes and knowledge in implicit evaluation. Cognit. Emot..

[bib39] Parker A.J., Woodhead Z.V.J., Thompson P.A., Bishop D.V.M. (2021). Assessing the reliability of an online behavioural laterality battery: a pre-registered study. Laterality.

[bib40] Peirce J., Hirst R., MacAskill M. (2022).

[bib41] Qi C., Fan X., Foxley S., Wu Q., Tang J., Hao W., Xie A., Liu J., Feng Z., Liu T., Liao Y. (2021). Structural imaging-based biomarkers for detecting craving and predicting relapse in subjects with methamphetamine dependence. Front. Psychiatr..

[bib42] Rehme A.K., Bey K., Frommann I., Mogg K., Bradley B.P., Bludau J., Block V., Sträter B., Schütz C.G., Wagner M. (2018). Selective attention to smoking cues in former smokers. Eur. Neuropsychopharmacol.

[bib43] Robinson T.E., Berridge K.C. (1993). The neural basis of drug craving: an incentive-sensitization theory of addiction. Brain Res. Rev..

[bib44] Rooke S.E., Hine D.W., Thorsteinsson E.B. (2008). Implicit cognition and substance use: a meta-analysis. Addict. Behav..

[bib45] Rosenberg H. (2009). Clinical and laboratory assessment of the subjective experience of drug craving. Clin. Psychol. Rev..

[bib46] Sawilowsky S.S. (2009). New effect size rules of thumb. J. Mod. Appl. Stat. Methods.

[bib47] Sayette M.A., Shiffman S., Tiffany S.T., Niaura R.S., Martin C.S., Schadel W.G. (2000). The measurement of drug craving. Addiction.

[bib48] Simon R., Snow R., Wakeman S. (2020). Understanding why patients with substance use disorders leave the hospital against medical advice: a qualitative study. Subst. Abuse.

[bib49] Tsai M.C., Chung C.R., Chen C.C., Yeh S.C., Chen J.Y., Lin C.H., Chen Y.J., Tsai M.C., Wang Y.L., Lin C.J., Wu H. (2021). An intelligent virtual-reality system with multi-model sensing for cue-elicited craving in patients with methamphetamine use disorder. IEEE (Inst. Electr. Electron. Eng.) Trans. Biomed. Eng..

[bib50] Westerhausen R., Samuelsen F. (2020). An optimal dichotic-listening paradigm for the assessment of hemispheric dominance for speech processing. PLoS One.

[bib51] Witkiewitz K., Bowen S. (2010). Depression, craving, and substance use following a randomized trial of mindfulness-based relapse prevention. J. Consult. Clin. Psychol..

[bib52] Wong K.M., Cloninger C.R. (2010). A person-centered approach to clinical practice. Focus.

[bib53] World Medical Association (2013). World Medical Association declaration of Helsinki: ethical principles for medical research involving human subjects. JAMA, J. Am. Med. Assoc..

[bib54] Zhao Q., Lu Y., Zhou C., Wang X. (2021). Effects of chronic exercise on attentional bias among individuals with methamphetamine use disorder. Psychol. Sport Exerc..

